The article "Research on CT Lung Segmentation Method of Preschool Children based on Traditional Image Processing and ResUnet" was published in 2022. Journal: Comput Math Methods Med.

# Research on CT Lung Segmentation Method of Preschool Children based on Traditional Image Processing and ResUnet

**DOI:** 10.1155/2022/7321330

**Published:** 2022-10-10

**Authors:** Zheming Li, Li Yang, Liqi Shu, Zhuo Yu, Jian Huang, Jing Li, Lingdong Chen, Shasha Hu, Ting Shu, Gang Yu

**Affiliations:** ^1^Department of Data and Information, The Children's Hospital Zhejiang University School of Medicine, Hangzhou 310052, China; ^2^Sino-Finland Joint AI Laboratory for Child Health of Zhejiang Province, Hangzhou 310052, China; ^3^National Clinical Research Center for Child Health, Hangzhou 310052, China; ^4^Polytechnic Institute, Zhejiang University, 866 Yuhangtang Rd, Hangzhou 310058, China; ^5^Department of Radiology, Children's Hospital, Zhejiang University School of Medicine, Hangzhou 310052, China; ^6^Department of Neurology, The Warren Alpert Medical School of Brown University, USA; ^7^Huiying Medical Technology (Beijing), Beijing 100192, China; ^8^The Children's Hospital Zhejiang University School of Medicine, Hangzhou 310052, China; ^9^National Institute of Hospital Administration, NHC, Beijing 100044, China

## Abstract

Lung segmentation using computed tomography (CT) images is important for diagnosing various lung diseases. Currently, no lung segmentation method has been developed for assessing the CT images of preschool children, which may differ from those of adults due to (1) presence of artifacts caused by the shaking of children, (2) loss of a localized lung area due to a failure to hold their breath, and (3) a smaller CT chest area, compared with adults. To solve these unique problems, this study developed an automatic lung segmentation method by combining traditional imaging methods with ResUnet using the CT images of 60 children, aged 0-6 years. First, the CT images were cropped and zoomed through ecological operations to concentrate the segmentation task on the chest area. Then, a ResUnet model was used to improve the loss for lung segmentation, and case-based connected domain operations were performed to filter the segmentation results and improve segmentation accuracy. The proposed method demonstrated promising segmentation results on a test set of 12 cases, with average accuracy, Dice, precision, and recall of 0.9479, 0.9678, 0.9711, and 0.9715, respectively, which achieved the best performance relative to the other six models. This study shows that the proposed method can achieve good segmentation results in CT of preschool children, laying a good foundation for the diagnosis of children's lung diseases.

## 1. Introduction

In recent years, the number of follow-up clinical diagnoses of respiratory diseases and the number of computed tomography (CT) lung applications has sharply increased. The proportion of CT lung examinations in children's radiological examinations has also increased, exceeding 25.12%. Lung CT is an important examination for ailments such as new coronary pneumonia, acute bronchial pneumonia, acute pneumonia, foreign bodies in the digestive tract, leukemia, sepsis, and atrial septal defect [1, 2]. However, because the image interpretation process is quite complex, and there may be differences in image evaluation and interpretation time among radiologists, many computer technologies are used to assist in the diagnosis of these diseases [3]. Computer-aided diagnosis of childhood lung diseases relies on accurate segmentation of the lung [4, 5], such as pneumonia detection [6], tuberculosis detection [7], and pulmonary nodule detection [8]. Lung segmentation can narrow the search range of lung lesion detection and reduce the interference of others, thereby effectively improving the accuracy of the diagnosis of other lung diseases.

So far, several methods have been developed for lung segmentation. Traditional image processing methods mainly include the following [9]: (1) threshold-based segmentation [10]. This method can be used to set threshold intervals and create binary partitions. Although it is faster, it does not consider the spatial distribution of image pixels and is sensitive to noise; thus, it is not ideal for the segmentation of images with litter gray-scale differences. (2) Region-based segmentation [11]. This method is fast and has a good segmentation effect under subtle attenuation changes. However, it often has some defects and underperforms in the segmentation of pathological boundaries. (3) Clustering-based segmentation [12–14]. This method can aggregate pixels with small gray value differences into the same category and divide an image into different regions through clustering. In a study by Wu et al. [15], three different differential edge operators were utilized to preprocess the images of 80 children with RMPP. The OA, FPR, and FNR of the RO were 0.935, 0.0427, and 0.0465, respectively. However, owing to the clustering algorithm, assignment of the initial point can be quite sensitive, resulting in different segmentations depending on the initialization. Deep learning algorithms are being implemented in medical image processing. In segmentation tasks, the Unet model [16] and its improved version [17–20] are one of the most widely used. They are applied to brain tumor segmentation [21, 22], lung nodule segmentation [23, 24], lung segmentation [25–28], liver segmentation [29], heart segmentation [30], etc. In addition to the 2D segmentation model, Çiçek et al. [31] proposed a 3DUnet that replaced the 2D convolution kernel with a 3D version and could learn the 3D information of the target. 3D-based segmentation includes multiscale 3D U-Nets [32], GA-UNet [33], and V. Net [34]. However, these 3D models could be limited by their computationally intensive design and limited effects on some segmentation tasks. Among the UNet-Zoo models, ResUnet is the more common model [35]. It introduces the Res module in ResNet into the Unet model by the rich skip connections within the network to facilitate information propagation. Using ResUnet as the referential background, different improvement models have been developed for different tasks [36–38]. Besides UNet-Zoo models, transformer-based models have also achieved good results in image segmentation tasks [39–41].

Although the methods mentioned above have been implemented in the study of adults' lung segmentation, they could not be used on preschool children's CT images due to issues such as (1) presence of artifacts caused by the shaking of children, (2) loss of a local area of the lung due to failure in holding their breath, and (3) smaller CT images chest area of preschool children. These characteristics are shown in Figure 1.

Based on current clinical and literature limitations, this study was aimed at building a lung segmentation by combining traditional imaging methods with ResUnet using preschool children on CT images with the hope that it could be used for diagnosing various lung diseases in the future. First, traditional image processing techniques were used to denoise, crop, and zoom the image, reduce the amount of calculation, and improve segmentation accuracy. Then, an optimized ResUnet model was used to segment the lungs of preschool children's CT images, whereby the unfit segmentation parts were removed through a case-based filter to improve the accuracy of the segmentation.

## 2. Algorithm Introduction

The proposed segmentation model consists of three parts: image preprocessing, improved ResUnet model, and case-based filtering. The method flowchart is shown in Figure 2.

### 2.1. Image Preprocessing

The image processing step consists of two parts. In the first part, a Gaussian filter is applied to the image to obtain a clearer CT image. In the second part, the image is cropped and resized based on the connected domain, allowing the model to learn more efficiently and quickly.

#### 2.1.1. Gaussian Filter

Considering that CT images can be affected by machine-related issues resulting in noises and blurriness due to the body shaking of children, for improved segmentation, the CT images are preprocessed using a Gaussian filter before segmentation, yielding relatively higher image qualities.

Gaussian filters are very effective low-pass filters in the space or frequency domains and are widely used in image processing. The 2D Gaussian function has rotational symmetry, and the smoothness of the filter is the same in all directions. Thus, a 2D Gaussian filter was used in this study, based on

(1) $$\begin{array}{c} G\left(x,y\right)=\frac{1}{\sigma \sqrt{2\pi }}{\text{e}}^{-\left({\text{x}}^{2}+{\text{y}}^{2}\right)/2\sigma^{2}}. \end{array}$$

Here, (*x*, *y*) represents the coordinates of pixels, and *σ* represents the width of the Gaussian filter. The width of the Gaussian filter determines the degree of smoothing. A larger *σ* suggests a wider band frequency of the Gaussian filter and better smoothness. However, if *σ* is too large, the image features could be blurred. To maintain clarity of the lung boundaries and remove associated noises for the subsequent segmentation, a *σ* value of 3 was selected.

#### 2.1.2. Image Cropping and Zooming

In the CT images of preschool children, the chest area only occupies less than 20% of the whole image. Therefore, many nontarget areas are present in the whole image, which increases the calculations and reduces the accuracy of the model. Thus, the algorithm used in this study first cuts off the original image based on the HU value of each organ in the CT image, then sets a threshold according to the gray value of the chest, performs the binarization operation on the image, forms the connected domain through the ecological opening operation, and then selects the circumscribed rectangular frame of the largest connected domain to crop the image to obtain a partial CT image containing only the chest area. Finally, all cropped CT images are zoomed to a uniform size of 256^∗^256. Compared with the original image size of 512^∗^512, this cropped and zoomed method reduces the model's amount of calculation and improves segmentation accuracy. The flowchart of this step is shown in Figure 3, and the corresponding effects are shown in Figure 4.

### 2.2. ResUnet Module

In this study, the ResUnet segmentation model was used as the segmentation method of preschool children's lung parenchyma. The model uses the Leaky-ReLU function, instead of the ReLU activation function, as the basic framework for the Unet network. A dropout strategy was implemented to improve the generalization of the model. To improve the detection rate of nodules and enhance the characteristics of the edges of nodules, the Res module is added to the Unet network model to increase the learning depth of the model. The lost part is simultaneously improved, which is conducive to improving the accuracy of the model. The overall network structure of the model is shown in Figure 5.

#### 2.2.1. The Res Module

To better integrate the global features of the images with their underlying features, in addition to the skip connection of the 3D Unet network in the encoding and decoding part of this study, for each convolution, the feature map before the convolution is combined with the one after the convolution. The feature maps are then connected, and the feature maps of the two parts of the concatenate are used as the output of this convolution. This operation extracts higher-dimensional features through convolutions while retaining the original dimensional features, thereby realizing an effective fusion of features at different scales and ensuring segmentation accuracy. The Res module is shown in Figure 6.

#### 2.2.2. Loss Improvement

To remove the influence of artifacts, Dice loss and local loss are combined as a new loss. Dice loss has better effects on class imbalance-related issues, while local loss has better effects on boundary-related issues. Dice loss comes from the Dice coefficient, which measures the degree of overlap between two samples. The measurement range is 0 to 1, and a Dice loss of 0 suggests a complete overlap. The calculation formula is as follows:

(2) $$\begin{array}{c} L_{\text{Dice}\left(e,f\right)}=1-\frac{2^{*}\left|e\cap f\right|}{\left|e\right|+\left|f\right|}, \end{array}$$

where *e* represents the ground truth and *f* represents the segmentation result.

Although Dice loss has better effects on class imbalance-related problems, its gradient oscillates greatly during the error backpropagation process and is unstable during the training process. The focal loss is a modification based on the cross-entropy loss function [17], which has good stability and also increases the loss value of hard negatives such as the transition area between the foreground and the background. The calculation formula is as follows:

(3) $$\begin{array}{c} L_{f}=\left\{\begin{array}{c} -\alpha {\left(1-y^{\prime }\right)}^{r}\log y^{\prime },\;y=1,\\ \left(1-\alpha \right)y^{\prime r}\log\left(1-y^{\prime }\right),\;y=0. \end{array}\right. \end{array}$$

Here, *r* represents a reduction in the loss of easy-to-classify samples to focus more attention on difficult and misclassified samples, and *ɑ* is used to balance the uneven ratio of positive and negative samples.

By combining the characteristics of focal loss and Dice loss, we hereby propose an improved focal loss based on the following formula:

(4) $$\begin{array}{c} L_{\text{all}}=\alpha \log L_{\text{Dice}}+L_{f}. \end{array}$$

Here, the purpose of the logarithmic function and *α* is used to balance the resulting size of the two loss functions. In this paper, *α* is set to 0.3.

### 2.3. Case-Based Filter

Despite the cropping and zooming in the first step, the positioning information of the lung area is not yet completely learned by the model. At the same time, because the model is based on 2D segmentation, the 3D information of the lungs is completely lost. Therefore, to obtain a complete case, after all the images are segmented by the model, a 3D domain connection is performed on the segmentation mask of the entire case to obtain multiple 3D volumes. Finally, according to the positioning information and the volume of the 3D body, the two larger 3D bodies, namely, the left and right pages of the lungs, are screened out. This process can effectively remove missegmentations in the pre-CT scan images and complement the loss parts of the lung due to issues such as the failure of the children to hold their breath. Segmentation after the base-cased filter is shown in Figure 7.

## 3. Experimental Results

### 3.1. Experimental Environment and Associated Parameters

The GE Optima CT660 machine was used to scan the lungs. Briefly, a child was placed in the supine position, with the head advanced, the arms held up, and the body placed in the center of the examination table. Before scanning, any metal ornaments and foreign bodies were removed to avoid artifacts. The scanning range started from the tip of the lungs to the bottom of the lungs. For children who did not cooperate with the examination procedures, a sedation was orally given using 5 mL of chloral hydrate syrup after a doctor's consultation. After the children went into a deep sleep, the CT lung examination was performed.

CT scanning parameters included a tube voltage of 100 kV and an automatic tube current of 30-300 mA, with a noise index of 12, pitch of 1.375 and rotation speed of 0.8 s/r. For the entire lung, the scan slice thickness and interval were both 5 mm, and the reconstruction slice thickness and interval of the lung window were both 0.625 mm.

To assess the performance of the proposed model, we conducted a method test using the chest CT images of preschool children. The LU-NA16chest CT dataset was used. We selected the thinnest CT images (0.4 mm), with each case having between 200 and 300 images after selection. All data were obtained from the Children's Hospital of Zhejiang University School of Medicine (Hangzhou, Zhejiang, China). The dataset included the CT images of 60 preschool children, of whom 33 were 0-2 years old, 23 were 3-4 years old, and 4 were 5-6 years old. Their age distribution is shown in Table 1.

All training, testing, and verification experiments were completed using the Ubuntu 16.04 server. The basic configuration was a CPU using Intel E5-1650 3.50 GHz, a 64G DDR4 memory, and an RTX 2080Ti graphics card. All annotation work was performed in the RadCloud (Huiying Medical Technology Co., Ltd., Beijing, China).

### 3.2. Evaluation Standard

In this study, the intersection over union (IOU), Dice coefficient (Dice), precision, and recall [8] were used as indicators to measure the performance of the algorithm. For this purpose, the following four variables were used: true positive (TP), true negative (TN), false positive (FP), and false negative (FN). The calculation formula of each index is as follows:

(5) $$\begin{array}{c} \text{IOU}=\frac{e\cap f}{e\cup f},\\ \text{Dice}\left(e,f\right)=2\frac{\left|e\cap f\right|}{\left|e\right|+\left|f\right|},\\ \text{Precision}=\frac{\text{TP}}{\text{TP}+\text{FP}},\\ \text{Recall}=\frac{\text{TP}}{\text{TP}+\text{FN}}, \end{array}$$

where *e* represents the gold standard and *f* represents the segmentation result.

### 3.3. Training Process

We divided the experimental data into three parts: training, validation, and test sets. In total, there were 48 cases in the training and validation sets, with 12,522 pictures, among which 11,270 pictures were for the training set and 1252 pictures for the validation set. The test set was made up of 12 cases and 3068 images. All models adopt RMSprop [42] as the optimizer with an initial learning rate of 0.001 and a training epoch of 10. All images were cross-segmented by two clinicians with at least 5 years of experience. For images with a segmentation error of less than 1% (assessed by two doctors), the gold standard was determined based on the average mask marked by the two doctors. The other images were marked as the final gold standard by the two doctors.

### 3.4. Result Analysis

The performance of our method based on the 12 cases of the test set is shown in Table 2.

As shown in Table 2, our method achieved an average accuracy of 0.9479, while the averages of Dice, precision, and recall on test set class are 0.9678, 0.9711, and 0.9715, respectively. We compare our method with Unet [16], Unet++ [17], Unet+++ [19], Attention-UNet [20], Swin-Unet [39], and Trans-Unet [40]. The segmentation results of different segmentation algorithms are shown in Table 3.

Table 3 shows that the IOU, Dice, and precision of the proposed method are higher than other algorithms by at least 1%. Unet+++ performs the best on recall, leading our method by 0.33%, but other metrics are all far from our method. For CT images of preschool children with artifacts and partial missing areas, the proposed method demonstrated good segmentation (Figure 8).

To better illustrate the value of building a preschool-specific lung segmentation model, we trained ResUnet on a publicly available adult lung database [43] containing 16,708 images and tested it on the test set used in this paper. It can be seen from the last row of Table 3 that the proposed model did not perform as well as the other models on the preschool lung segmentation task. The possible reason is that the images on the adult lung cancer dataset are relatively clear, and the lungs account for a higher proportion of the image, where these features are different from those of children. More details on the performance of the Unet model applied to adult lung segmentation on our test set are shown in Table 4.

In summary, our method achieves the best segmentation performance on CT images of preschool children.

## 4. Discussion

In this study, we proposed a novel model based on traditional image algorithms and ResUnet to segment lung from CT scans of preschool children. On the validation set containing 12 cases, our method achieved Dice, precision, and recall of 0.9678, 0.9711, and 0.9715.

Lung segmentation is one of the important foundations for intelligent diagnosis of many lung diseases, and accurate segmentation can effectively improve the performance of diagnostic models. In literature [44], Primakov et al. first extracted the lungs to allow the model to focus on the ROI prior to the detection and segmentation of non-small-cell carcinomas. In literature [45], the authors summarize the application of AI in the diagnostic dilemma of pulmonary nodules over the past 20 years. The first step of all methods is lung segmentation and then the detection or segmentation of pulmonary nodules. Due to the epidemic of the COVID-19, the classification and lesion detection of COVID-19 has become one of the research hotspots, and the first step in all research is also lung segmentation [6, 46–49]. However, lung segmentation studies on CT of preschool children are still relatively rare.

The first step of this paper is to collect CT images of 60 children aged 0-6 years. Compared with the adolescents and adults, preschool children have smaller lung, which brings greater challenges to lung segmentation. As shown in Tables 2–4, our experiments also demonstrate that if the model trained on the adult database is directly used to segment the lungs of CT images of preschool children, its performance is almost lower than that of all segmentation models trained on the preschool database. On the preschooler validation set, the Dice score of the ResUnet model trained on the adult database [43] is 3 percentage points lower than that of the ResUnet model trained on the preschooler database. This result suggests the necessity of designing a segmentation algorithm for preschooler lung segmentation.

Second, we noticed that many literatures only use one of traditional image algorithms [10–15] or deep learning [26, 50, 51], failing to fully combine the advantages of both. For the challenges existing in the lung segmentation of preschool children, we combined traditional image algorithms and deep learning as solutions. Because preschool children's lung is small, this paper used the traditional image algorithm based on connected domain to extract the body area first. The benefit of this step is to remove extraneous areas such as the bed, thereby normalizing the CT images of children of different ages and concentrating the lung in the middle of the image. Then, we used a deep learning model which is good at segmentation tasks to complete the initial segmentation. Finally, we optimized the segmentation results through traditional image algorithms. Through the effective combination of different algorithms, our method achieves good performance in the lung segmentation task of preschool children.

Finally, we compared with the current mainstream methods, including models based on Unet and Transformer. The results obtained by our proposed model are superior compared to other models.

It should be noted that this study has examined only on the dataset of our hospital, and the cases included in this study are relatively small, and our model needs to be verified and optimized on other data. Secondly, on the basis of accurate lung segmentation, it is necessary to further study the intelligent diagnosis of lung diseases in preschool children.

In conclusion, this method combining traditional image algorithms and deep learning models can accurately segment the CT lung of preschool children, which provides a good foundation for subsequent studies such as classification of childhood pneumonia and detection of childhood pulmonary tuberculosis.

## 5. Conclusions and Prospects

Accurate lung segmentation of the CT scans of preschool children is of great significance to accurately and timely detect and analyze lung nodules and pneumonia in real-world clinical settings. This study proposes an automatic lung segmentation method that combines traditional imaging methods with ResUnet using the CT images of preschool children. First, Gaussian filtering was used to denoise the image, followed by image ecology operations to crop and zoom the CT images. Then, an optimized ResUnet model was used to segment the 2D image, and unfit segmentation parts were removed through a case-based filter to improve the accuracy of the segmentation. According to the experimental results, the proposed segmentation method could correctly segment most CT images of the investigated preschool children and extract relatively complete lungs. Compared with other deep learning models and traditional image processing methods, the proposed method could reduce the adverse effects of child hyperactivity on segmentation and improve the accuracy and speed of lung segmentation. In addition, using the proposed method, the segmentation of the lungs was closely related to specific clinical applications. Comparison with other segmentation methods showed that they could not be uniformly applied to the chest CT images of preschool children. In future studies, we will continue investigating other lung segmentation methods to achieve higher segmentation accuracy.

## Figures and Tables

**Figure 1:** Chest CT image of a preschool child with (a) artifacts (labeled as 1), (b) loss of a local area of the lung (labeled as 2), and (c) adult lungs image which has larger lung area than children).

**Figure 2:** Algorithm flowchart of the proposed segmentation.

**Figure 3:** Image cropping and zooming of the model.

**Figure 4:** Illustration of the (a) original CT images (size, 512^∗^512) and (b) the corresponding cropped and zoomed images (size, 256^∗^256).

**Figure 5:** The overall structure of the ResUnet module.

**Figure 6:** The overall layout of the Res block.

**Figure 7:** Comparisons before and after case-based filter. The red parts represent the segmentation result. (a) Segmentation results before case-based filter. (b) Segmentation results after case-based filter.

**Figure 8:** The proposed method versus gold standard method and other methods.

**Table 1:** Dataset.

Ages (years)	Train set	Test set
0-2	28	5
3-4	17	6
5-6	3	1

All	48	12

**Table 2:** Performance of the test set.

Case no.	IOU	Dice	Precision	Recall
1	0.9552	0.9754	0.9733	0.9782
2	0.9602	0.9794	0.9802	0.9789
3	0.9543	0.9746	0.9805	0.9699
4	0.9604	0.9786	0.9788	0.9791
5	0.9599	0.9783	0.9789	0.9792
6	0.9442	0.9664	0.9608	0.9809
7	0.9559	0.9753	0.9786	0.9753
8	0.9578	0.9778	0.9873	0.969
9	0.8874	0.9084	0.907	0.9481
10	0.9444	0.9647	0.9736	0.966
11	0.95	0.9717	0.9717	0.9753
12	0.9449	0.9636	0.9829	0.9587

Average	0.9479	0.9678	0.9711	0.9715

**Table 3:** Segmentation results of different segmentation algorithms.

Method	IOU	Dice	Precision	Recall
Unet	0.934	0.9553	0.9561	0.9625
Unet++	0.9338	0.9543	0.9493	0.9699
Unet+++	0.9359	0.9568	0.9468	0.9748
Attention-UNet	0.9257	0.9482	0.9424	0.9673
Swin-Unet	0.8738	0.917	0.8998	0.949
Trans-Unet	0.9364	0.9569	0.9611	0.9592
Proposed method	0.9479	0.9678	0.9711	0.9715
ResUnet (adult)	0.9163	0.9368	0.9351	0.9451

**Table 4:** Performance of the Unet model applied to adult lung segmentation on our test set.

Case no.	IOU	Dice	Precision	Recall
1	0.9226	0.9436	0.9357	0.9535
2	0.9305	0.9497	0.9481	0.9514
3	0.9164	0.9397	0.937	0.9434
4	0.9291	0.9477	0.9413	0.9558
5	0.9248	0.9441	0.9438	0.9494
6	0.9172	0.9391	0.9283	0.9562
7	0.9261	0.9459	0.9436	0.9505
8	0.9295	0.9483	0.9507	0.9476
9	0.8561	0.8766	0.8764	0.909
10	0.912	0.9333	0.9365	0.9415
11	0.9158	0.9394	0.9331	0.9497
12	0.9151	0.9345	0.9462	0.9329

Average	0.9163	0.9368	0.9351	0.9451

## Data Availability

The data used to support the findings of this study are available from the corresponding author upon request.
